This article has been retracted.

# Emotional Cognitive Expression in Lacquer Colors Based on Prior Knowledge

**DOI:** 10.1155/2022/1151676

**Published:** 2022-08-30

**Authors:** Ping Wei

**Affiliations:** Shanghai University, Shanghai Academy of Fine Arts, Shanghai 200444, China

## Abstract

Since lacquer painting first appeared in the world of art, research into it has grown steadily. People have developed a keen interest in modern lacquer painting as a result of the extensive study of lacquer culture in both domestic and international academic circles. Many artists and art enthusiasts have contributed significantly to the study and research of lacquer painting and have made helpful attempts at modern lacquer painting. But it is challenging to describe the emotion that a lacquer painting's color conveys. This paper presents a decision-making framework for emotional cognitive learning based on the theory of emotional cognitive evaluation because there are relatively few researchers who have specifically studied the relationship between the creation of lacquer paintings and emotions and because there are also few research materials and documents for reference. The assessment of an emotional state is the central component of this framework. The observation module in the model framework is used to gather the emotional data that the lacquer painting expresses. The issue of emotional expression in lacquer painting is resolved by the emotional evaluation system, which combines the preprocessed information with prior knowledge to evaluate. The importance of affective cognitive expression in lacquer painting and the necessity of affective computing in the fields of machine learning and decision control is obtained on the basis of discussing the research status and content of affective cognition and affective computing. The efficiency of expression was increased by 1.3 percent as a result.

## 1. Introduction

After being nurtured, modern lacquer painting has been continuously influenced by the artistic trend in the background of great art, which catalyzed the new state of lacquer painting art. Modern lacquer painting constantly enriches itself based on its own unique materials and techniques, and the number of artists in the continuous growth and development is also increasing, which makes lacquer painting have great room for improvement in expressiveness and emotional expression. The picture is not only an image but also a spatial representation of an illusion. By drawing on the plane, the painter flexibly uses a variety of visual and spatial information to draw objects that do not exist in reality but can be perceived. This construction from objective space to cognitive space is a unique skill of human beings. What people say about painting as the art of creating optical illusions is this kind of spatial representation. There are no boundaries in art, and art is even more interlinked. For the art of painting, the best performance is the coolness of the techniques or the strong basic skills, and the works of real artistic value must have certain visual effects and artistic appeal.

Emotional cognition [1] is the resonance of the emotions that a person or thing produces. A few articles explore the process, specificity, and meaning of this contribution to literary experience. Alcorn and Neill used historical evidence to argue that the affective influence of a native son restructures the cognitive practice of segregation empowerment [2]. Niu and Huang conducted research on topics such as sentiment analysis and cognition. His research goal was to analyze people's perceptions, emotions, evaluations, and attitudes toward entities and attributes. Word-level sentiment cognition has become an important topic in sentiment analysis. Compared with the traditional method, the engine has the advantages of fast processing speed and low occupancy rate, making up for the disadvantages of the previous method, which is time-consuming and computationally complex [3]. Changes in fatty acids were analyzed by using a paired sample *t*-test. Zhang et al. believed that cognitive and affective behaviors need to be measured by the Executive Function Behavior Rating Scale-Adult Test, State-Trait Anxiety Scale, and 3-item Loneliness Scale [4]. Davila et al. participated in an interactive task that assessed their ability to adapt to the expression of positive emotions. The results showed that a woman's romantic capacity was positively correlated with her and her partner's ability to express positive emotions, even controlling for relationship satisfaction. She discussed what it means to understand the expression of positive emotions in young couples and the need to enhance romantic capacity to facilitate it [5]. Although these documents have well explained the importance of emotional cognition, they have not been combined with the art of lacquer painting to illustrate, lacking a certain pertinence.

Lacquer colors are often used in the field of painting. Ewa has demonstrated his research through various architectural activities, and he took such action as necessary to help dispose of buildings of historical significance while preserving the value of the original buildings [6]. Silverman provided a long-term study based on ethnography. Colors and paintings that evoke landscapes were analyzed from the history of myth, totemism, the aesthetic value of movement, irreducible dialogues about the becoming of the universe, and ontological principles of water change [7]. Since most paintings change color over time, Loon et al. wanted to learn more about what the paintings looked like in the first place and what they did in his paintings. He also provided new information on the distribution and composition of trace elements in paints. Paint reconstruction was performed to study the effect of different percentages on the overall color [8]. The color of the lacquer painting is a very important part of the painting, but there is still a lack of research on emotional cognition.

Modern lacquer painting differs from other types of art, despite the limitations imposed by the unique properties of lacquer. In addition to production methods, material selection, and other components, lacquer painting creation also carries significant symbolic meaning. The unique artistic effect of lacquer painting is achieved because the painter is frequently constrained by the subject and content, the material and craftsmanship, and other factors during the creation process. The following aspects of this paper reflect its innovations:. The interactive system with emotional capabilities is simulated within the model framework. Facial expression recognition, emotional state assessment, emotional cognitive decision-making, emotional behavior, etc. make up the majority of it. Compared to the earlier model framework, it adds a system that is more comprehensive.

## 2. Emotional Cognitive Approaches

### 2.1. Affective Cognitive Model

The prospect theory and reinforcement learning theory, which emphasise the importance of influencing emotion in decision-making and neurally-based human decision-making behavior, are extensions and integrations of the existing theories that make up the affective cognitive model. The affective cognitive model postulates that the presumed decision-making preferences are primarily derived from the subjective experience in analogous past situations and can accurately predict the future affective effect of the choice. The predictive model [9] is a goal-directed reflex process, while the experience-based model is typically a reflective, associative, and automatic process, as shown in Figure 1.

According to the assumption, affective cognitive decision-making only occurs in a single cognitive state during a specific time window, and the observation model provides information on this state. The cognitive reward model is *M*_*AM*_(*a*′), and the cognitive state transition model formula is as follows:

(1) $$\begin{array}{c} Pn\left(a^{\prime }|a,f\right). \end{array}$$

The emotional model formula is as follows:

(2) $$\begin{array}{c} Pn\left(d^{\prime }|a^{\prime },d\right). \end{array}$$

The emotion conversion model formula is as follows:

(3) $$\begin{array}{c} Pn\left(d^{\prime },d|d_{p},a,f\right)=\sum_{i=1}^{\left|A\right|}Pn\left(d^{\prime }|a^{\prime }=i,d_{p}\right)Pn\left(a^{\prime }=i|a,f\right). \end{array}$$

The affective cognitive decision-making models formulas are given as follows:

(4) $$\begin{array}{c} Q_{AN}\left(a,b,f\right)=Q_{\text{ext}}\left(a,f\right)+Q_{\text{int}}\left(a,b,f\right), \end{array}$$

(5) $$\begin{array}{c} Pn\left(f=k|a,b\right)\frac{\text{exp}\left(\alpha Q_{AN}\left(a,b,f\right)\right)}{\sum_{l=1}^{\left|F\right|}\text{exp}\left(\alpha D_{AN}\left(a,b,l\right)\right)}. \end{array}$$

Here *α* is the inverse temperature of the selection strategy.

### 2.2. Affective Cognitive Decision

The essence of the process of an emotional agent interacting with people in an unknown environment is a mapping process that the agent establishes the state space of the external environment and the behavior space of the emotional agent by continuously accepting the extrinsic and intrinsic rewards from emotional cognition [10]. Therefore, it is necessary to define the emotional state of the agent receiving the reward.

**Definition 1 .**

The emotional state space in an emotional agent is FI, as shown in the following formula:

(6) $$\begin{array}{c} FI=\left\{FI_{1},FI_{2}\right\}. \end{array}$$

**Definition 2 .**

The emotional agent accepts the emotional state space in the external environment as *FX*, as shown in the following formula:

(7) $$\begin{array}{c} FX=\left\{FX_{1},FX_{2},FX_{3},FX_{4}\right\}. \end{array}$$

**Definition 3 .**

The action space of the emotional agent is B, as shown in the following formula:

(8) $$\begin{array}{c} B=\left\{B_{1},B_{2},B_{3},B_{4}\right\}. \end{array}$$

The emotion-cognitive decision-making algorithm operates in a self-loop, initialising the affective agent's extrinsic emotion probability distribution at the same time as initialising the affective agent's inner emotional state space set FI in the emotional agent as “happy, unhappy,” the external emotional state space set FX as “joy, sadness, fear, and anger,” and the cognitive state as “juvenile.”

The observation module allows the emotional agent to learn about the interactor's emotional state, and it then updates its external emotion probability distribution, as shown in the following formula:

(9) $$\begin{array}{c} ef_{i}=Pn\left(e=i|a,{\text{ef}}_{\text{old}}\right)=\sum_{j=1}^{\left|E\right|}Pn\left(e=i,e_{\text{old}}=j|a,{\text{ef}}_{\text{old}}\right). \end{array}$$

To the input layer of the neural network is sent the probability distribution of the current emotional state. The intrinsic cognitive reward value *U*_int,*a*_ is calculated using the *M* function in the hidden layer of the neural network, as shown in the following formula:

(10) $$\begin{array}{c} U_{\text{int},a}=M_{AR}\left(a,j\right). \end{array}$$

Intrinsic emotional reward value *U*_int,*ei*_ is given as follows:

(11) $$\begin{array}{c} U_{\text{int},ei}=M_{EIR}\left(\text{ef},a,j\right)=\sum_{j=1}^{\left|E\right|}epM_{EIR}\left(i,a,j\right). \end{array}$$

The intrinsic reward value *U*_int_ is calculated as follows:

(12) $$\begin{array}{c} U_{\text{int}}=\chi_{A}\left(j\right)\times U_{\text{int},a}+\chi_{E}\times U_{\text{int},ei}. \end{array}$$

By calculating the maximum intrinsic reward value output by the neural network, the emotional agent selects the corresponding emotional behavior decision *j* to execute, as shown in the following formula:

(13) $$\begin{array}{c} Pn\left(j=k|a,b\right)=\frac{\text{exp}\left(\alpha Q_{DM}\left(a,b,j\right)\right)}{\sum_{l=1}^{\left|D\right|}\text{exp}\left(\alpha Q_{DM}\left(a,b,l\right)\right)}. \end{array}$$

After executing decision *j*, the observation module obtains the extrinsic reward *y*_*ext*_, and then uses the model *Y*_ext_ to update the extrinsic reward, as shown in the following formula:

(14) $$\begin{array}{c} Y_{\text{ext}}\leftarrow \left(1-\lambda \right)R_{\text{ext}}\left(a,j\right)+\lambda r_{\text{ext}}. \end{array}$$

### 2.3. Artificial Neural Network

Artificial intelligence theories that emulate biological information processing models include fuzzy set theory, neural networks [11–13], and evolutionary algorithms. Without taking into account the role of human perceptual thinking in the process of information processing, all of these theories are realised by rational and logical thinking. The biological information processing system is a complex network made up of interconnected meridian elements, and the artificial neural network primarily mimics this biological information processing mechanism in nature.  Figure 2 illustrates the three categories of input units, output units, and hidden units, which are used to classify the different types of neuron processing units used in artificial neural networks.

The input-output relationship of the artificial neuron model formulas are as follows:

(15) $$\begin{array}{c} M_{j}=\sum_{i=1}^{n}w_{ji}d_{i}-\beta_{j}=\sum_{i=0}^{n}w_{ij}d_{i}\left(d_{o}=\beta_{j},w_{j0}=-1\right), \end{array}$$

(16) $$\begin{array}{c} h_{j}=f\left(m_{j}\right). \end{array}$$

Among them, *β*_*j*_ is the threshold; *w*_*ij*_ is the connection weight coefficient. The output transformation functions that are often used are as follows:

(1) Proportional function (linear function)
  (17) $$\begin{array}{c} f\left(m\right)=m. \end{array}$$
(2) Symbolic function
  (18) $$\begin{array}{c} f\left(m\right)=\left\{\begin{array}{c} 1\left(m\geq 0\right),\\ -1\left(m<0\right). \end{array}\right. \end{array}$$
(3) Hyperbolic function
  (19) $$\begin{array}{c} f\left(m\right)=\frac{1-e^{-\delta s}}{1+e^{-\delta s}}. \end{array}$$
(4) S line function
  (20) $$\begin{array}{c} f\left(m\right)=\frac{1}{1+e^{-\delta s}}. \end{array}$$

## 3. Experimental Deconstruction of Emotional Cognition

### 3.1. Overview of Emotional Cognition in Lacquer Painting

#### 3.1.1. Overview of Lacquer Painting

Visual art includes painting. The viewer can receive the most immediate visual experience and stimulation from materials. Different materials evoke various emotions in the viewer. It is important to remember that the material serves as the lacquer painting's carrier. The reasons modern lacquer painting flourishes in the garden of art are largely due to its distinctive aesthetic approach, distinctive aesthetic traits, and distinctive material performance, which is comparable to the relationship between landscape painting and rice paper, ink and oil painting, and canvas and pigment.

A piece of art is always a composite made up of various materials. Material art's texture and the specifics of artistic expression are closely related. The material used in contemporary lacquer paintings includes both the actual lacquer and any texture or texture effect that is produced by the material. The surface feature of an object is its texture. A hierarchy of space will appear visually due to the material's surface's various colors and patterns. It has unique expressiveness as a modelling element. Modern people constantly develop new texture aesthetics as well as endless natural textures that they perceive in everything in nature. For the final visual performance of space, the material is a necessary and significant component, as illustrated in Figure 3.

Traditional western painters construct the picture primarily using the focus perspective method in order to give the illusion of three-dimensional space and then combine expression techniques like color, light, and shade to accurately depict the space. The best technique used by western painters to express focal perspective is their attempt to produce three-dimensional space paintings. The best technique used by western painters is the expression of focal perspective. They want to be able to produce three-dimensional space images. The use of the scientific focus perspective method is the most important modelling factor to express the three-dimensional and three-dimensional sense of the object on the two-dimensional plane [14], as shown in Figure 4.

#### 3.1.2. Emotional Cognitive Process

The primary function of the process of emotional cognition is to alter people's emotions in response to outside stimuli. It is also the emotional experience and emotional behaviorbehavior that people's attitudes toward the objective world give rise to in their hearts. One feature that sets humans apart from the current generation of intelligent machines is our capacity for emotion. Calculating variables that are connected to emotions, stimulated by emotions, or that can affect emotions in computers or machines is referred to as affective computing. Through studies on emotion theory, neurology, and physiology, psychologists, cognitive scientists, and physiologists have made an effort to systematically explain the mind-body processes and relationships of emotion [15].

Emotional experience is closely related to personal life and the evaluation of things. According to the theory of emotional cognitive evaluation, emotion is the emotional experience that an individual produces when he evaluates a subjectively important event. Since different individual emotions are related to psychology, belief, and the external environment, the final emotional state is closely related to the individual's cognition and subjective evaluation of stimuli [16]. The evaluation process of the emotional cognitive evaluation theory is shown in Figure 5.

The process of emotional cognition is mainly the process of emotional changes of people under external stimuli, which is the emotional experience and emotional behavior produced in the heart by people's attitudes toward the objective world.

#### 3.1.3. Emotional Cognitive Evaluation Model

Since the non-negligible role of emotion and cognition in people's daily lives and employment is being increasingly recognised by researchers in the fields of cognitive psychology and artificial intelligence, more people are studying the cognitive evaluation theory of emotion, and there are numerous common and representative cognitive evaluation theories (such as OCC and Roseman). The OCC emotion model was the first model made for computer use. They are even quantified using mathematical formulas and theories for computer calculations. The theory of affective cognitive evaluation has never been mathematically quantified in computers before, but OCC is the first to do so [17]. According to cognitive evaluation theory, it is possible to distinguish between various emotional states using a number of evaluation standards. As a result, using different evaluation standards will produce different fundamental emotion classification methods and outcomes, as shown in Table 1.

Roseman's evaluation theory believes that evaluation can be performed according to the criteria of the interaction of specific elements, so it also has a systematic framework for defining evaluation criteria and performing calculations. In the Roseman cognitive evaluation model, the evaluation factors of emotion are divided into five factors: accident, motivation, possibility, control, and cause. Then, according to these five emotional evaluation factors, the basic emotions are given: surprise, happiness, relief, sadness, and depression. According to the cognitive evaluation theory table, five emotional evaluation factors and five basic emotions are given in the structure diagram [18].

#### 3.1.4. Extraction of Emotion Types

There are 20 basic emotions in the OCC model and 15 basic emotions in the Roseman model. They are too complicated in the actual operation process, so six types of emotional states are adopted. Because most facial expression recognition systems now use five emotions, which is also an important way to reflect personal emotions, the later research on facial expression recognition is almost always based on the facial expression coding system to build a facial expression recognition model, as shown in Figure 6.

There are only four basic expressions of fear, joy, sadness, and anger in the overlapping part of the model, which is not surprising. This is so because this fundamental expression type does not produce compound responses and has little to do with cognitive processes. It is awkward to directly use the emotion types to calculate the emotional state because the model only includes 20 fundamental emotions and the emotion types are too complex. The model's division of emotions into five categories of expressions makes it simple to identify facial expressions. Figure 6 displays the classification of emotions. By maintaining the integrity of expressions when dealing with a small number of emotional states, it is possible to increase the naturalness and harmony of interactions between machines and people [19].

### 3.2. Static Experiment of Emotional Cognition

#### 3.2.1. Experimental Mode

The subjects were 30 users with severe or moderate red-green dysesthesia with normal or corrected visual acuity and no other visual abnormalities.

#### 3.2.2. Experimental Devices

In the experiment, a laptop with a 10-inch monitor was used to display digital colors, and a laptop with Internet access was used to collect and record experimental data online.

#### 3.2.3. Experimental Materials

All single-color, two-color, and three-color digital colors required for the experiment were made into digital color cards.

The ten test single colors are all one color. Cognitive experiments with 70 different color combinations using two color produce results with clearly discernible color. Since the background and foreground color issues were not present in the emotional association experiment, or because the two color combinations that were alternated between the background and foreground colors were regarded as repeated color combinations, the repeated color combinations were then removed, leaving 60 color combinations. Then, these color schemes were chosen by five subjects who had moderate to severe red-green dysesthesia, and those who responded similarly to emotional associative stimuli were put into one category. One color combination from each category was chosen as a representative for testing after the results of the selection of the five subjects were integrated. As a result, the experiment was run more effectively and the subject's operation was simplified, which had little impact on the experiment's outcomes. 30 two-color color combinations total were eventually obtained for the emotional association experiments. The results of the two-color cognitive experiment, that is, the 140 colors mentioned earlier, were used to create a three-color color combination that was easily recognisable. The In the same way, these three-color combinations were chosen and summarised by five individuals who had moderate to severe red-green dysesthesia, yielding a final 30 three-color color combinations for the emotional association experiment.

The recorded questionnaires used by the subjects to select emotional association words were prepared. The recorded questionnaire of the positive test was that the title was the color picture number, and the options were the generalized emotional association vocabulary. The recorded questionnaire was uploaded to the questionnaire star for the subjects to choose online during the experiment.

#### 3.2.4. Experimental Procedure

First, the subjects were given a brief explanation of the overall goal and methodology of the entire experiment. As in the cognitive experiment, the subject was checked for abnormal red and green perception prior to the experiment if they were a new participant who had not taken part in the cognitive experiment. This was done to ensure the accuracy of the experiment. A subject could take the test if they complied with the moderate-to-severe requirements. After that, the experiment was declared to have begun, and the forward experiment was run first. The subjects were shown single-color, two-color, and three-color color swatches sequentially on a laptop with a 10-inch display. The subjects were instructed to carefully consider the emotional associations that each color card evoked while viewing it, and then select 1-2 (up to 2) words from the list that they felt most closely matched. The subjects of the experiment filled out a questionnaire on another networked notebook, which was used to facilitate the statistics of the data. The subjects were instructed to take a break every 15 to 20 minutes to prevent visual fatigue.

A reverse test was then conducted after that. The test takers clicked on the questionnaire star next to the recorded questionnaire of the reverse test, which corresponded to each word with an emotional association. The color that best matched the association described by the word was chosen and numbered from the digital color card displayed on a laptop with a 10-inch monitor. Three different color schemes—one, two, and three—were used for the experiments. The subjects were instructed to take a break every 15 to 20 minutes to prevent visual fatigue. The entire static experiment process took about an hour.

#### 3.2.5. Analysis of the Results

In this experiment, the order of the concentration of the subjects' choice of emotional association words for each color card was taken as the basis for judging the emotional association generated by the color or color combination. For the experimental errors caused by the abnormal degree of red-green color perception and fatigue, the influence on the experimental results was reduced by detecting the abnormal color vision and letting the subjects rest before the experiment. The main errors in the current experiment were that the degree of abnormal color vision was different and the emotional association sensitivity of individuals to color stimuli was different. The experimental results combined the results of the forward experiment and the reverse experiment, and then the common experimental results were found. The experimental results of individual cases with large deviations were removed, and the vocabulary with the highest concentration of the positive and negative experimental results at or above was obtained as the emotional association generated by the color or color combination. The details are shown in Table 2. The same as the cognitive experiment results, the color HSB values in Table 2 represent the interval value of the color [20].

Since the emotional association of color stimuli is a highly subjective experiment, not all vocabulary can concentrate on corresponding color results. Especially for two-color and three-color, it is more difficult. Therefore, there are some words in the two-color and three-color results that cannot lead to significant color results. In addition, the same as the results of the cognitive experiment, each color interval contains several colors. That is, each color interval represents many colors, so the above experimental results can represent a wider range of colors.

### 3.3. Dynamic Experiment of Emotional Cognition

Due to the particularity of digital color, this study innovatively added the study of dynamic color to the emotional experiment. The difference between the emotional association and static color produced in the transformation of color was studied. The experimental process is as follows:

#### 3.3.1. Experimental Subjects

The subjects were 30 users with severe or moderate red-green abnormal vision who participated in the static color experiment with normal or corrected vision and no other visual abnormalities.

#### 3.3.2. Experimental Device

In the experiment, a laptop with a 10-inch monitor was used to display digital colors, and a laptop with Internet access was used to collect and record the experimental data online.

#### 3.3.3. Experimental Materials

All the two-color color combinations and three-color color combinations used in all the static emotional association experiments were made into transformed gif dynamic pictures with gif production software, which were used for dynamic color emotional association experiments.

Similar to the static emotional association experiment, the recorded questionnaires used by the subjects to choose emotional association words were prepared. The dynamic experiment only conducted a positive test. That is, the questionnaire was recorded as the title and the color picture number. The option was the generalized emotional association vocabulary, and the recorded questionnaire was uploaded to the questionnaire star for the subjects to choose online during the experiment.

#### 3.3.4. Experimental Procedure

Similar to the static experiment, the subjects were first given an overview of the overall goal and methodology of the study. The experiment then got underway. The subjects were exposed to turn-by-turn displays of two- and three-color dynamic gif colorcolor-switching color cards on a laptop with a 10-inch monitor. The subjects had to carefully consider the emotional associations associated with each color card as they changed, as opposed to the static colors, and select one or two words from the provided vocabulary that were most similar to those associations. The experimental data was filled out on the questionnaire by the subjects and uploaded beforehand on another networked notebook to simplify the statistics of the data. Every 20 minutes, the subjects were instructed to take a break to prevent visual fatigue. The dynamic experiment took about 50 minutes to complete. It was discovered following the experiment that the subjects' experimental data had been successfully uploaded.

#### 3.3.5. Analysis of the Results

As in the static experiment, in this experiment, the subject's order of the concentration of emotional association words selected by each color card was used as the basis for judging the emotional association generated by the color or color combination. In the experimental results, words with a concentration degree of at or above were selected as the emotional associations generated by the dynamic color combination, which were the same as the previous results. The specific results are shown in Table 3.

As mentioned above, the emotional association experiment for color stimuli was a highly subjective experiment. Compared with the static experiment, the dynamic color experiment required the subjects to feel the sensitivity of color stimuli more subtly, which was more difficult. Therefore, there are also some words that could not yield significant color results. In addition, as in the previous experimental results, each color interval contained several colors. That is, each color interval represented multicolor verification of barrier-free color design methods and practical and experimental results. The above experimental results can represent a wider range of colors.

### 3.4. Experimental Results and Deconstruction of the Improved Algorithm

A row and column of squares were programmed in the programming environment, and several tiny squares (obstacles) were placed there to create a small maze. After that, the agent was programmed to find the target by automatically navigating past all of the maze's obstacles. Through this maze experiment, the improved algorithm was validated.  Figure 7 [21] displays the algorithm's experimental findings.  Figure 7 illustrates how, after numerous failed attempts to find the target in the maze, the agent is able to successfully navigate around the obstacles encountered in the search process.

The starting point was set at *T* = 90. The neural network that realised the *Q* function took into account whether there were any obstacles to the left, right, up, and down, and the output layer represented four different left, right, up, and down actions [22]. The experimental outcomes of locating the target in the maze using the conventional algorithm were compared in order to more clearly see how effective the improved algorithm was, as shown in Figure 8.

The parameters in the two algorithms were identical, and the results of the traditional algorithm experiment and the improved algorithm experiment were compared when the agent located the target in the maze [23]. The average reward received by the emotional agent after locating the target using the conventional algorithm and the improved policy algorithm is compared in Figures 8 and 9, along with the number of trials required to locate the target successfully [24].

## 4. Conclusions

In the modern era of diversified art, the creation of lacquer painting should integrate the past and the present, allowing traditional methods to be painted, and also allowing people to combine Chinese, western, and modern methods to paint. From the figurative to the abstract, from the west to China, from the traditional to the modern, the artists are free to gallop. Modern lacquer painting presents a diversified trend in space expression, so its future development has more possibilities. Actually, no matter whether it is the artistic style or the creative concept, it can add luster to the spatial performance of modern lacquer painting. The unique artistic style created by modern painters is an important symbol of their success. Artists' individuality is the life of a work of art, and their character, spiritual quality, way of thinking, and aesthetic taste all affect the creation of the work. If every artist creates with his own concepts and standards, an art world full of different styles and full of interest can be created, which reflects the importance of emotional expression. Some progress has been made in the application of affective computing in human-computer interaction systems with emotion. However, due to the different perspectives and methods of emotion modelling, there are still limitations in emotion modelling. Meanwhile, emotion research faces many challenges in the acquisition of emotional information, the transmission of emotional states, and the expression of emotional behaviors. But overall, emotional cognition in lacquer painting still improved expression efficiency by 1.3%.

## Figures and Tables

**Figure 1:** Basic framework of the emotion model.

**Figure 2:** Artificial neural network.

**Figure 3:** Traditional lacquer artwork.

**Figure 4:** Lacquer painting in western painting language.

**Figure 5:** Emotional cognitive evaluation process.

**Figure 6:** Five basic expression categories.

**Figure 7:** Experimental results of the agent finding the target.

**Figure 8:** Comparison of traditional (left) and improved (right) algorithms.

**Figure 9:** Comparison of trial times for traditional (left) and improved (right) algorithms.

**Table 1:** Five emotional evaluation factors and five basic emotional structures.

	Unexpected	Possibility	Motivation	Reason	Control bit
Surprise	Unexpected				
Happy			Promote		
Gratified		Sure			
Sad		Disgust		Caused by the environment	
Suppressed					Low control

**Table 2:** Results of single-color, two-color, and three-color static color emotion association experiments.

Emotional association vocabulary	Single-color	Two-color	Three-color
New	H0S0B0	H50S0B80	H230S0B0
Old	H50S0B0	H230S80B40	H50S0B0
Cold	H50S0B80	H50S0B20	H50S0B40
Warm	H50S0B0		

**Table 3:** Results of single-color, two-color, and three-color static color emotion association experiments.

Emotional association vocabulary	Single-color	Two-color	Three-color
New	H20S0B0	H50S0B80	H80S0B0
Old	H80S0B0	H500S0B40	H230S0B0
Positive	H50S0B0	H50S0B20	H40S0B40
Negative	H50S0B0	H2300S0B0	H50S0B40

## Data Availability

The data used to support the findings of this study are available from the corresponding author upon request.
